This article has been retracted.

# Study on Intelligent Traditional Chinese Medicine Fumigation for Treating Lumbar Intervertebral Disc Herniation Based on Medical Big Data Mining

**DOI:** 10.1155/2022/4658192

**Published:** 2022-10-13

**Authors:** Jirong Zhao, Ping Zhang, Guodong Gao

**Affiliations:** ^1^Department of Spinal Surgery, Affiliated Hospital of Gansu University of Chinese Medicine, Lanzhou, Gansu 730000, China; ^2^Gansu University of Chinese Medicine, Lanzhou, Gansu 730000, China; ^3^College of Electrical and Information Engineering, Lanzhou University of Technology, Lanzhou, Gansu 730050, China

## Abstract

With the improvement of the traditional Chinese medicine fumigation (TCMF), more and more people are studying lumbar intervertebral disc herniation (LIDH) by TCMF. In order to clarify the thermodynamic mechanism of TCMF to LIDH and provide a model reference for individualized diagnosis, the lower control system is compiled by the microprocessor, and the upper control system is compiled by computer technology of VB. In this new system, the medical information of patients is recorded in the databases by the upper control system, and clinical diagnosis and treatment experience are packaged in the lower control system. The simulation results and clinical examples show that the new control system of TCMF has better clinical efficacy for LIDH patients, which not only effectively improves the pain symptoms of LIDH patients but is also economical and safe.

## 1. Introduction

LIDH is a common disease in orthopedics. It causes low back pain or leg pain, seriously endangers the health of patients, and even leads to disability [1, 2]. LIDH not only seriously affects the quality of life of patients but also increases the economic burden of patients [3]. As an important part of traditional medicine, traditional Chinese medicine fumigation has a definite effect in the treatment of LIDH. It can not only improve the pain symptoms of patients with LIDH, strengthen the automatic congestion and phagocytosis of the organism, and promote cell growth and regeneration, but it is also economical and safe. However, the efficacy of traditional Chinese medicine fumigation is affected by multiple factors such as temperature and treatment time. How to dynamically adjust the fumigation time and treatment temperature according to the patient's physical signs is the key point in individualized clinical treatment plan [4, 5].

TCMF is one of the treasures of Chinese medicine. It uses the physiological characteristics of the skin to ensure that the drug is absorbed through the surface of the skin and enters the blood circulation to achieve the therapeutic effect [6]. The earliest document of TCMF is the “Fifty-two Prescriptions for Diseases,” which has been developed for thousands of years. At present, the research of TCMF focuses on the integration of traditional treatment methods and clinical case discussion [7]. Quantitative mathematical description and unified scientific norms have not yet been formed. Temperature is a macroscopic expression of energy transfer. Factors such as patient signs, outdoor temperature, and fumigation formula interact with fumigation temperature. Based on this, the establishment of the traditional Chinese medicine fumigation temperature model has important research value for inheriting and developing traditional Chinese medicine.

According to the data recorded in clinical cases, it is proved that temperature has significant clinical effects on the treatment of lumbar disc herniation by TCMF. The paper observes 300 clinical cases and points out that temperature has a significant influence on the treatment effect in different courses of treatment [8]. Since FU-LC published “Why our Western-trained doctors should learn traditional Chinese medicine” in the “Chinese medical journal” in 1955, the research of traditional Chinese medicine fumigation has gradually attracted the attention of scholars. Due to the difference in analysis methods, TCMF is still tracking learning and clinical records. The traditional Chinese medicine fumigation treatment process inherited the unique Chinese “analogy” mode of thinking. It is a way of thinking that seeks common ground in differences [9, 10]. In the process of diagnosis and treatment, a large number of oral treatment experiences and vague concepts (such as pain and slight pain) cannot be analyzed by mechanism modeling. Therefore, using artificial intelligence methods to identify the process of clinical diagnosis and treatment experience of famous traditional Chinese medicine doctors is the way to solve the above problems. The diagnosis model of TCMF based on the Yinger learning algorithm is shown in Figure 1.

Temperature is an important treatment parameter in traditional Chinese medicine fumigation. The experienced orthopedic doctor dynamically adjusts the fumigation temperature according to the patient's physical signs. This is the process of human brain judgment and reasoning. In the fumigation process, the patient's physiological process and the energy transfer process affect each other and restrict each other, which makes industrial temperature control methods unable to effectively model and control such temperature systems. Therefore, the use of abundant clinical resources to carry out TCMF temperature system modeling and control research is not only of important research value for in-depth analysis, mining, and utilization of clinical resources, inheritance, and development of TCMF but also for saving energy consumption and improving human health. It has research significance.

The rest of this paper is organized as follows: Section 2 discusses the patient's information and traditional Chinese drug fumigation control system, followed by the thermodynamic model of fumigation in Section 3, simulation experiment on TCMF is discussed in Section 4, and Section 5 concludes the paper with summary and future research directions.

## 2. Patients' Information and Research Methods

The illustration of the traditional Chinese drug fumigation machine is the type of machine that is DXZ-1, and it has been used 5 years. The mixture of water and Chinese herbal medicines are homogenized in the container for 30–50 minutes. The doctor treats the lumbar disc herniation with steam generated by boiling medicinal herbs.

### 2.1. Patient Information Database Analysis

It is important to observe the symptoms of patients when working with machine. There are lots of medical mobile data throughout the therapy. So, the traditional Chinese drug fumigation system consists of the host computer and slave computer two-level system. The medical mobile data are transmitted from slave computer system to host computer system [11, 12]. Users can enter the upper control system through registration or authorization.

The system consisted of permission login interface, user basic information interface, user medical history information interface, course interface, the real-time temperature interface, and the evaluation interface. The system can be operated in Windows XP, Windows Vista, and Windows7-Windows 11. In the upper system, patient personal information and treatment parameters can be recorded here, such as patient's gender, age, course of disease, heat source output power, prescription, fumigation time, medical history, outdoor temperature, and efficacy level. By analyzing that information, the mechanism of traditional Chinese medicine fumigation treatment can be further explained. Traditional Chinese medicine fumigation is one of the treasures of traditional Chinese medicine. It is one of the effective nonsurgical methods for the treatment of lumbar disc herniation. Traditional Chinese medicine fumigation uses the physiological properties of the skin to absorb the drugs through the skin surface and enter the blood circulation to achieve the therapeutic effect.

The user first comes to the welcome interface and then clicks the “click to enter the system” button, and the user will come to the login interface which can register an account. After the user successfully logs in to the account, the user will enter the next interface, which is the upper temperature monitoring system of the fumigation machine. This interface can communicate with the lower computer. After the serial port is successfully opened, it can receive and send relevant temperature information in real time, including accepting the lower real-time temperature, upper and lower limit temperatures, and setting the fumigation time set by the user. The set upper and lower limit temperature is transmitted to the lower position. This operation interface can also quickly enter the temperature control interface, where the upper computer can control the working state of the lower fumigation machine (for example, when the temperature is lower than the lower limit, the heating plate is heated. On the other hand, when the temperature is higher than the upper limit, the heating plate stops heating), and the upper position will have a corresponding indicator light to keep the temperature within a constant range. The patient basic information is recorded in the host computer system to database for next date analysis.

### 2.2. Treatment Process Information Database Analysis

During the treatment process, the temperature is recorded by temperature sensor that is enclosed in a protective well in the slave computer system, and then the message is transmitted to the host computer system. The temperature and treatment time of the fumigation process can be displayed on this page in real time.

There are about 600 LIDH patients in our hospital every year, and about 65% of patients can use Chinese medicine fumigation to relieve pain. This article selects 650 patients with LIDH who are treated in our hospital from March 2020 to October 2021 as the research object to record all medical information. Some patients' information is shown in Table 1. The inpatient office inputs patient's basic information on the host computer and offers hospitalization record in the database. The course of treatment is determined by seasoned doctors.

In Table 1, A is qi-stagnancy and blood stasis, B is cold and dampness, C is moist heat arthralgia, *D* is deficiency of the liver and kidney. In medical evaluation methodology, 4 denotes healing, 3 is tangible results, 2 means valid, and 1 is invalid.

### 2.3. Lower Control System Analysis

The temperature control system takes PIC16F877 as the main controller which automatically executes different working conditions according to expert experience database. The upper and lower limits of the temperature can be set from upper and lower control systems. The DS18B20 temperature sensor can measure the temperature in real time. The PIC16F877 devices come in 40-pin packages, and it has a 13 bit program counter capable of addressing an 8K *x* 14 program memory space. On the other hand, it has 8K *x* 14 words of FLASH program memory. The solid-state relay is a part of the control module. When the measured temperature value is lower than the set lower limit, the heating drive circuit works to heat the liquid. On the other hand, when the temperature reaches the set range, the heating drive circuit is disconnected, and the constant temperature is maintained. The stirring motor operates to stir the liquid medicine, and the heat stored in the liquid medicine is released rapidly through stirring. When the temperature exceeds the set range, the heating plate and stirring motor do not work, and the system starts to alarm.

## 3. Thermodynamic Model of Fumigation

### 3.1. Fuzzy Neural Network Topology Structure

The dynamic fuzzy neural network is shown in Figure 2, and it includes 5 layers: input layer, membership function layer, if layer, then layer, and output layer.

Layer 1: every node in layer 1 represents an input.

(1) $$\begin{array}{c} X={\left[x_{1}\cdots x_{n}\right]}^{T}\text{.} \end{array}$$

Layer 2: every node in layer 2 represents a membership function, which is in the form of Gaussian.

(2) $$\begin{array}{c} \mu_{ij}\left(x_{i}\right)=e\text{.} \end{array}$$

In this, *i*=1, ⋯, *n*, *j*=1, ⋯, *r*.*μ*_*ij*_is the membership function of the input variable*x*_*i*_,*σ*_*j*_is the center of the Gaussian membership, and *c*_*ij*_ is the width of the Gaussian membership.

Layer 3: every node in layer 3 represents a possible rule for fuzzy rules.

(3) $$\begin{array}{c} \varphi_{j}=e\text{,} \end{array}$$

in which, *i*=1, ⋯, *n*, *j*=1, ⋯, *r*

Layer 4: each node in layer 4 represents the then

(4) $$\begin{array}{c} \phi_{j}=\frac{\varphi_{j}}{\overset{r}{\underset{k=1}{\sum }}\varphi_{k}}\text{,} \end{array}$$

in which, *j*=1, ⋯, *r*.

Layer 5: each node in layer 4 represents the output variable as a weighted summation of incoming signals.

(5) $$\begin{array}{c} y\left(x\right)=\frac{\sum_{k=1}^{r}\left[\left(a_{k_{0}}+a_{k_{1}}x_{1}+\cdots +a_{k_{n}}x_{n}\right)e\right]}{\sum_{i=1}^{r}}\text{,} \end{array}$$

in which, *k*=1, ⋯, *r*.

So

(6) $$\begin{array}{c} y_{j}\left(X\right)=\overset{m}{\underset{j=1}{\sum }}\omega_{ij}\mu_{A_{1}^{i_{1}}}\left(x_{1}\right)\mu_{A_{1}^{i_{2}}}\left(x_{2}\right)\cdots \mu_{A_{1}^{i_{n}}}\left(x_{n}\right)/\overset{m}{\underset{j=1}{\sum }}\mu_{A_{1}^{i_{1}}}\left(x_{1}\right)\mu_{A_{1}^{i_{2}}}\left(x_{2}\right)\cdots \mu_{A_{1}^{i_{n}}}\left(x_{n}\right)\text{,}\\ =\overset{m}{\underset{j=1}{\sum }}{\omega_{ij}R}_{j}/\overset{m}{\underset{i=1}{\sum }}R_{i}\text{,}\\ =\overset{m}{\underset{j=1}{\sum }}\omega_{ij}{{\bar{R}}_{j}}_{i}\left(X\right)\text{.} \end{array}$$

Let basis function*h*(*X*)as follows:

(7) $$\begin{array}{c} h\left(X\right)=\frac{\overset{n}{\underset{i=1}{\prod }}\mu_{A_{i}^{j}}\left(x_{i}\right)}{\overset{m}{\underset{j=1}{\sum }}\left(\overset{n}{\underset{i=1}{\prod }}\mu_{A_{i}^{j}}\left(x_{i}\right)\right)}\text{.} \end{array}$$

Then

(8) $$\begin{array}{c} h\left(X\right)=\frac{\overset{n}{\underset{i=1}{\prod }}\mu_{A_{i}^{j}}\left(x_{i}\right)}{\overset{m}{\underset{j=1}{\sum }}\left(\overset{n}{\underset{i=1}{\prod }}\mu_{A_{i}^{j}}\left(x_{i}\right)\right)}\text{,}\\ =\frac{\exp\;\left[-\left(\sum_{i=1}^{n}{\left(x_{i}-c_{ij}\right)}^{2}/2\sigma_{ij}^{2}\right)\right]}{\overset{m}{\underset{j=1}{\sum }}\exp\;\left[-\left(\sum_{i=1}^{n}{\left(x_{i}-c_{ij}\right)}^{2}/2\sigma_{ij}^{2}\right)\right]}\text{,}\\ =\frac{\exp\;\left[{\left\|X-C\right\|}_{2}^{2}/2\sigma_{ij}^{2}\right]}{\overset{m}{\underset{j=1}{\sum }}\exp\;\left[{\left\|X-C\right\|}_{2}^{2}/2\sigma_{ij}^{2}\right]}\text{.} \end{array}$$

So

(9) $$\begin{array}{c} Y=\overset{m}{\underset{j=1}{\sum }}\omega_{ij}h\left(X\right)\text{,}\\ =WH=f\left(X\right)\text{.} \end{array}$$

From the slave computer system, we can see that the system has 9-dimensional inputs and 1 output. The inputs are as follows: patient's gender, age, course of disease, heat source output power, prescription, fumigation time, medical history, outdoor temperature, and the efficacy level. On the other hand, *n*=9.

### 3.2. Fuzzy Neural Network Algorithm

**Step 1 .**

Initial parameter settings

The parameters of network have not been determined when the first set of data is input, so the data should be made as follows:

(10) $$\begin{array}{c} C_{1}=X_{1}\Leftrightarrow c_{11}=x_{1}\left(t_{1}\right),\cdots ,c_{91}=x_{9}\left(t_{1}\right)\text{,}\\ \sigma_{1}=\frac{E}{3}{\left[1\cdots 1\right]}^{\tau }\Leftrightarrow \sigma_{11}\left(t_{1}\right)=0.334,\cdots ,\sigma_{91}=0.334\text{,}\\ W_{1}=\omega_{11}=\omega =D\left(X_{1},X_{d}\right)=\sqrt{{\left\|X_{1}-X_{d}\right\|}^{2}.} \end{array}$$

Here, *E* is the universe of input.*σ*_*j*_is the center of the Gaussian membership, and *c*_*ij*_ is the width of the Gaussian membership. The system has 9-dimensional inputs and 1 output, so*i*=1, ⋯9, *j*=1.

**Step 2 .**

Membership function

If the number of rules is too small, the system cannot completely contain the input-output state space. On the contrary, if the number of rules is too large, it will increase the complexity of the system and poor generalization ability. Therefore, the output error is an important factor in determining whether new rules should be added.

Let

(11) $$\begin{array}{c} E_{i}=D\left(X_{i},X_{d}\right)\times \left\|{\hat{y}}_{i}-y_{i}\right\|\text{.} \end{array}$$

In this paper, the system is a multiple input single output system.

Get

(12) $$\begin{array}{c} E_{i}=D\left(X_{i},X_{d}\right)\cdot \left|{\hat{y}}_{i}-y_{i}\right|\text{.} \end{array}$$

From (12), the initial error of learning is large, and the error gradually decreases as the learning progresses. The error is ${\hat{y}}_{i}$which is initial, and there is no one fuzzy rule in learning spaces before the first data are read. When the first data are entered, one rule is set up, and the width of membership functions benchmark is adjusted based on the probability theory of 3*σ*.

So the

(13) $$\begin{array}{c} D_{i0}=\frac{E}{3}\text{.} \end{array}$$

(14) $$\begin{array}{c} D_{i}=D\left(X_{i},X_{d}\right)\times \frac{E}{3}\text{,} \end{array}$$

in which, *E* is the universe of new input.

Figure 3 is the membership function surface. The *x*-axis represents the input domain and *X*=[−1,1]. The *y*-axis represents *σ*_*ij*_, and it ranges from 0.131 to 0.5. The *z*-axis represents the degree of membership, and it ranges from 0 to 1.

Figure 4 is the membership function width change trend surface. The *x*-axis represents the input domain and *X*=[−1,1]. The *y*-axis represents *σ*_*ij*_, and it ranges from 0.131 to 0.5. The *z*-axis represents the degree of membership, and it ranges from 0 to 1. As the learning progresses, the membership width gradually decreases.

All membership function surfaces are shown in Figure 5. The *x*-axis represents the input domain and *X*=[−1,1]. The *y*-axis represents *σ*_*ij*_, and it ranges from 0.131 to 0.5. The *z*-axis represents the degree of membership, and it ranges from 0 to 1. It is clearly evident from Figure 5 that the shape of the membership function is relatively smooth at the beginning of learning, which meets the requirements of using a low-resolution blur subset in a large area of error. When the width of the membership function changes, the number of rules also changes, and the upper limit can be seen to be 7 according to the fuzzy subset distribution, which coincides with the theoretical analysis results of the pruning technique.

**Step 3 .**

Parameter identification of membership function

Get the optimal function as

(15) $$\begin{array}{c} J=J\left(Y^{*}\right)=\overset{k}{\underset{l=1}{\sum }}{\left[d_{l}-Y\left(X_{l}\right)\right]}^{2}+\lambda {\left\|DY^{*}\right\|}^{2}\text{,}\\ =\overset{k}{\underset{l=1}{\sum }}{\left[d_{l}-HW\right]}^{2}+\lambda {\left(DY^{*},DY\right)}^{2}\text{,}\\ =\overset{k}{\underset{l=1}{\sum }}{\left[d_{l}-HW\right]}^{2}+\lambda \varpi^{T}G_{0}\varpi \text{.} \end{array}$$

Here, *d*=*ϖ*=(*d*_1_, ⋯*d*_*n*_)^*τ*^.

Let optimal function *J*be minimum when *ϖ*is adjusted.

So, we can get the rules as follows:

(16) $$\begin{array}{c} \omega ={\left(H^{\tau }H+\lambda H\right)}^{-1}H^{\tau }d\text{,}\\ \omega \left(k+1\right)=\omega \left(k\right)-\eta \left[\left(H^{\tau }H+\lambda H_{0}\right)\omega \left(k\right)-H^{\tau }d\right]\text{.} \end{array}$$

Here, *η*is set by system response time.

In this paper, Figure 6 is the flow chart of our proposed algorithm.

## 4. Case Analysis and Data Statistics

This article selects 500 cases among 2000 patients LIDH who are treated in our hospital from March 2020 to October 2021. Then, let 300 cases as the training set, 200 cases as the cross validation set, and 100 cases as the text set. We record all medical information by Section 2.2. Through the experimental results, it can be observed that the fumigator outside temperature is changed with time; felicitously adjusting heater output power can not only cure the patients but also reduce energy consumption.

Temperature is an important therapeutic parameter in traditional Chinese medicine fumigation [13, 14]. Experienced orthopedic surgeons dynamically adjust the fumigation temperature according to the patient's physical signs, which is a process of human brain judgment and reasoning. The wind speed of outdoor is shown in Figure 7. The *x*-axis represents the fumigation time, which is measured in minutes. The *y*-axis represents the wind speed, which ranges from 18 to 30 kilometers per second.

Figure 8 shows the three-dimensional treatment course curve. The *x*-axis represents the fumigation time, which is measured by minutes. The *y*-axis represents the fumigation temperature, which ranges from 0 to 10 degrees Celsius. The *z*-axis represents output power, which ranges from 400 to 1600 watt. In Figure 8, A denotes local, B denotes nerve root, C denotes spinal cord, *D* denotes vertebral artery, and *E* denotes sympathetic. It is clearly evident from Figure 8 that different treatment methods should be used to treat different types of patients.

The fumigation space temperature can be affected by the physical parameters of the space due to the presence of conduction and convection heat exchange. When we adjust fumigation liquid dosage, the space temperature can be reobtained to target status by the controller. The space temperature of TCDF has no effect on external disturbance by the controller of the algorithm in Section 3.3, as shown in Figure 9. The temperature is set to a constant value of 40 degrees Celsius. It is clearly evident from Figure 9 that the temperature at the location of the heat source is the highest. Due to the existing conduction and convection heat exchange methods, the temperature of the fumigation space is closely related to the physical parameters of the space. Although the system is subject to external disturbances, it has no effect on the spatial temperature distribution. On the other hand, the temperature controller based on the new system has good knowledge extraction ability, and the robustness of the control system is high.

Using this medical mobile data management clinical work, Figure 10 is the lumbar MR of hospitalization number 22578 after 2 days. The variable structure dynamic fuzzy neural network was used to control and predict relevant parameters of TCMF process. Different from the previous dynamic fuzzy neural network, the structure of the variable structure dynamic fuzzy neural network studied in this paper is not preset but dynamically changed. There are no fuzzy rules before learning, and the fuzzy rules of the network are gradually formed through learning. The number of fuzzy rules obtained by this method does not show an exponential growth trend with the increase of the number of inputs. This kind of network has a significant effect on the modeling and knowledge extraction of TCM fumigation temperature control system. In addition, the network structure is compact, which effectively avoids the phenomenon of overfitting.

The fumigation time and fumigation temperature were dynamically adjusted according to the clinical feedback of the patient. The patient was discharged after 18 days of treatment, and the clinical symptoms were significantly relieved at this time. The MR of return visit after 8 months is shown in Figure 11. The left posterior protrusion completely disappeared, and the symptoms of the patient are completely relieved.

Temperature control strategies for patients with small probability will be studied in the future. The data involved in the research of the thesis are obtained through clinical experiments. Due to the randomness of the patient's condition, the data of some special cases will be excluded as unclean data during data preprocessing. In the future, the improvement of the algorithm should be added to the research on the temperature control in small probability cases. Due to the heat conduction during the drug boiling process, the water in the drug liquid mixture evaporates, and the liquid concentration changes dynamically with time, which limits the application of the established hydrodynamic mode. In the next step, the existing temperature system model should be improved and optimized to strengthen system functions, deeply mine spatial information, improve clinical treatment effects, and reduce energy consumption.

## 5. Conclusion

TCMF is a common method for the treatment of lumbar disc herniation, and it is widely used in clinical practice because of its remarkable curative effect, low cost, and small side effects. However, the temperature is constrained by multiple factors, resulting in the inability to fully exploit and utilize the rich clinical experience and practical accumulation of the past dynasties, which not only hinders the digital development of TCMF but also causes a lot of clinical data mining work that cannot be carried out normally. In order to solve this problem, the new system of TCDF uses an intelligent control and database method to research on data mining and mechanism model analysis. So, this new diagnosis and treatment method can be clinically analyzed and promoted, and this has laid theoretical and technical support for the promotion of self-employed treatment of LIDH.

## Figures and Tables

**Figure 1:** Diagnosis model of TCMF.

**Figure 2:** Model of dynamic fuzzy neural network.

**Figure 3:** Membership function surface (*c*_*ij*_=0).

**Figure 4:** Membership function width variation trend surface.

**Figure 5:** All membership function surface.

**Figure 6:** Flow chart of our proposed algorithm.

**Figure 7:** The wind speed of outdoor.

**Figure 8:** Three-dimensional curve of power, time, and temperature.

**Figure 9:** Space temperature (1200 seconds).

**Figure 10:** Lumbar MR (2 days).

**Figure 11:** Lumbar MR (8 months).

**Table 1:** Patients' information.

Hospitalization number	22578	10112	35689	34869	42556	46887	50236	51226	55328	58962
Sex	Male	Female	Male	Female	Male	Female	Male	Female	Male	Male
Age	47	43	39	41	58	35	55	62	39	48
Type	A	D	C	B	C	B	B	B	A	B
Beginning temperature of steam (Celsius degrees)	45	46	47	48	49	46	47	49	48	47
Finishing temperature of steam (Celsius Degrees)	42	45	45	50	50	45	48	47	49	49
Average temperature of lumbar (Celsius degrees)	38	37	41	40	38	39	41	42	42	42
Time of fumigation(minute)	27	33	28	36	30	25	35	29	31	38
Total time of therapy(day)	18	14	10	11	16	13	15	18	16	20
Curative effect	3	2	1	4	2	4	3	4	3	4

## Data Availability

The simulation experiment data used to support the findings of this study are available from the corresponding author upon request.
